# To Explore the Application of PDCA in Hemodialysis Center and Its Effect on the Maintenance of Internal Fistula

**DOI:** 10.1155/2022/7380632

**Published:** 2022-07-20

**Authors:** Xiaomei Su, Yihong Cui, Zunguo Pu, Yaqing Zhou

**Affiliations:** ^1^Department of Nephrology, Affiliated Hai'an Hospital of Nantong University, Hai'an County, Nantong City, Jiangsu Province 226600, China; ^2^Department of Critical Care Medicine, Affiliated Hai'an Hospital of Nantong University, Hai'an County, Nantong City, Jiangsu Province 226600, China

## Abstract

**Background:**

The survey found that in recent years, with the incidence of chronic kidney disease (CKD) increasing, some patients with CKD even progressed to end-stage renal disease. Luckily, progressive hemodialysis technology and nursing level can improve the quality of life and prognosis of patients.

**Objective:**

To explore the application of plan-do-check-adjust (PDCA) cycle in the management of nurses in hemodialysis center and its effect on the maintenance of internal fistula in patients.

**Methods:**

In this study, a randomized controlled trail (RCT) was used to select 90 patients who underwent maintenance hemodialysis in the hemodialysis center of our hospital from January 2018 to June 2021 as objects. They were divided into a PDCA group (with PDCA nursing management) and routine group (with routine nursing management) by random number table with each of 45 cases for 6 months to compare the differences of the internal fistula complications, internal fistula maintenance quality, patients' microinflammatory state, and satisfaction with nursing, as well as nursing staff's operational and theoretical performance between the two groups.

**Results:**

There was no significant difference in CRP, IL-1, TNF-*α*, and IL-6 levels between the two groups before intervention (*P* > 0.05); after that, these levels in the PDCA group were lower than those in the routine group, with statistically significant difference (*P* < 0.05); before intervention, there was no statistically significant difference in the qualification rate of blood flow, the awareness rate of health education, and the incidence of nursing defects between the two groups (*P* > 0.05); after that, the qualification rate of blood flow and the awareness rate of health education among nurses in PDCA group were higher than those in routine group, while the incidence of nursing defect accidents in the PDCA group was lower than that in routine group, and the differences were statistically significant (*P* < 0.05); before intervention, there was no significant difference in the complication rate between the two groups (*P* > 0.05); after that, the complication rate of the PDCA group was lower than that of the routine group, and the differences were statistically significant (*P* < 0.05); after intervention, the theoretical assessment and practical skills assessment scores of the PDCA group were higher than those of the routine group, and the differences were statistically significant (*P* < 0.05); after intervention, the nursing satisfaction of the PDCA group was higher than that of the routine group, and the differences were statistically significant (*P* < 0.05).

**Conclusion:**

The application of PDCA approach in the management of nurses in hemodialysis centers can effectively improve the quality of internal fistula management and improve the practical and theoretical level of nurses, as well as reduce the microinflammation of patients.

## 1. Introduction

Hemodialysis is the main treatment for patients with acute and chronic renal failure and uremia. In the course of treatment, patients need to establish vascular access, and arteriovenous fistula is the first choice. This vascular access has the advantages of small trauma and high safety, but the cycle is long. It may require repeated internal fistula puncture, which easily causes a series of complications such as bleeding at the puncture point, local skin hematoma, failure, and infection and affects the therapeutic effect of patients [1, 2]. Good arteriovenous fistula is the key to determine the quality of dialysis and quality of life. Hemodialysis patients may lose confidence in treatment and affect prognosis due to long treatment cycle and irreversible course [3, 4]. Clinically, whether some effective intervention measures can be used to improve the maintenance quality of arteriovenous fistula in hemodialysis patients and ultimately improve the quality of dialysis is considered, but there are few relevant literatures [5, 6].. Studies have shown that the correct nursing is an important factor affecting the survival period of fistula [7, 8].. Traditional nursing methods lack systematicness and pertinence. In recent years, PDCA cycle training has been gradually introduced into clinical practice, but there is no clinical report on its role in improving the quality of hemodialysis patients [9]. In this study, the application of PDCA circulation was emphasized, and the influence on the maintenance of internal fistula during hemodialysis was analyzed in the nursing training.

### 1.1. Core Tips

The quality of care after hemodialysis is related to the recovery of patients' prognosis. PDCA cycle method is a new type of nursing management method. At present, the PDCA cycle method has not been well popularized. In this study, a randomized controlled study was used to compare the effects of PDCA nursing management mode and routine nursing management mode on the maintenance of internal fistula and the quality of hemodialysis in hemodialysis patients.

## 2. Materials and Methods

### 2.1. General Information

In this study, RCT was used to select 90 patients who underwent maintenance hemodialysis in the hemodialysis center of our hospital from January 2018 to June 2021 as objects. They were divided into a PDCA group (with PDCA nursing management) and routine group (with routine nursing management) by random number table with each of 45 cases.

Inclusion criteria were as follows: (1) patients from 19 to 75; (2) patients who received maintenance hemodialysis in the hemodialysis center of our hospital for 2-3 times a week; (3) all the underlying diseases the patients had were chronic renal failure (CRF); (4) patients who have received dialysis treatment for more than 6 months; and (5) the research program needs to meet the requirements of the medical ethics expert group of our hospital, and informed consent needs to be signed both by patients and their families.

Exclusion criteria were as follows: (1) patients with underlying diseases of coagulation system; (2) patients with malignant tumors; (3) patients with infectious underlying diseases (like abdominal infection, pulmonary infection); (4) patients who are being attacked by cerebrovascular disease, heart disease, etc., in recent 3 months; (5) patients with mental or cognitive dysfunction; and (6) patients with hematological diseases.

### 2.2. Dialysis Therapy

The autologous arteriovenous fistula vascular access was used for dialysis. The surgical methods included the side to end anastomosis and end to end anastomosis of the head vein and radial artery. The Fresenius hemodialysis machine and the cellulose triacetate membrane with a membrane area of 1.4 m2 were used for the hemodialysis treatment. The dialysis fluid was bicarbonate, and the dialysis water was reverse osmosis water. The related parameters in dialysis were as follows: 500 mL/min; blood flow: 200-300 mL/min; dialysis time: 4 h, 3 times a week; and anticoagulant medicine: low molecular heparin.

### 2.3. Intervention Measures

The patients in the routine group accepted routine nursing mode, evaluating positively to observe internal fistula, recording the changes of basic signs, and making sure of the sterile state during the treatment. Pay attention to communicating with patients and their family members, maintaining quiet and suitable department environment, and formulating scientific diet plan for the patients. Give them systematic guidance after being discharged from the hospital.

The PDCA group adopted PDCA nursing management mode, including (1) first, set up a nursing team, including 2 attending physicians and 4 nurses. All of them should first learn the theoretical knowledge of PDCA cycle management mode and systematically grasp the nursing points. (2) Plan: the head nurse should take the lead in formulating nursing goals, that is to say, extending the life of arteriovenous fistula and reducing the incidence of complications. After the target task is determined, the members of the group are required to develop a set of nursing process based on clinical experience and network resources and to develop a standard nursing process of arteriovenous fistula after discussion. (3) Do: (1) the head nurse should make an overall arrangement of training and designate the responsibility nursing system. Each nurse need to manage 2-6 patients, achieving the entire 8-hour working time for a continuous nursing in the day. In addition to the management of patients, nurses should also carry out education and training for the patients' families, so that they can master nursing knowledge, in order to take care of patients at home for improving the quality of the recovery period. (2) During the puncture of internal fistula, nurses need to assess the skin performance of patients. Nurses should strengthen the inspection of patients during dialysis for the changes in their signs. Stop bleeding, and band the puncture point with sterile dressings and elastic bandages after dialysis. (4) Check: the head nurse needs to regularly investigate and evaluate the nursing work and record the maintenance of fistula and skin performance of patients in detail as well as process them in time. (5) Adjust: forecast events that have occurred or have not happened yet for adjusting the nursing plan in time.

### 2.4. Observation Indicators and Detection Methods

The serum inflammatory factors: CRP, IL-1, TNF-*α*, and IL-6, were detected and compared between the two groups.

A total of 5 mL fasting venous blood was collected separately during the intervention and after that, and the serum was collected after centrifugation. The levels of TNF-*α*, IL-1, and IL-6 were detected by ELISA. The CRP level was detected by immunoturbidimetry, with the kit purchased from Roche, USA.

The incidence of subcutaneous hematoma, fistula blockage, infection, steal syndrome, and swelling hand syndrome was compared between the two groups. The evaluation of internal fistula maintenance quality mainly includes the qualification rate of blood flow (internal fistula blood flow velocity>150 mL/min), the awareness rate of patients on health education, and the incidence of nursing defect accidents.

The theoretical examination and practical skills of nursing staff were compared between the two groups by tests. Fifty theoretical examination questions were randomly selected from the nursing assessment library of our hospital for 2 points per question; while practice skills were mainly examined from the selection of puncture site, fistula observation, complication and stress treatment, and other aspects with a total of 100 points [10].

The average score of patient's satisfaction with nursing was calculated according to the subjective survey of patients with a total of 100 points. Patients can do the survey on the basis of their feelings during treatment. The higher the score, the more their satisfaction with nursing; being equal or greater than 90 points means he is very satisfied with nursing service, 80-89 points means satisfactory, 70-79 points means general, and less than 70 points means unsatisfactory [11].

### 2.5. Statistical Treatment

In this study, the serum CRP, IL-1, TNF-*α*, and IL-6 levels and other measurement indexes of patients were tested by normal distribution, which were in line with the approximate normal distribution or normal distribution, expressing as ($\bar{x}\pm s$). The *t* test was used for comparison between the two groups; nongrade count data were expressed by percentage (qualified rate of blood flow, awareness rate of patients on health education, incidence of nursing defect accidents, etc.), and statistical analysis was performed by the *χ*^2^ test; nonparametric test method was used for comparison of grade count data (nursing satisfaction classification), with professional SPSS21.0 software for data processing, test level *α* = 0.05.

## 3. Results

### 3.1. Comparison of Baseline Data between the PDCA Group and Routine Group

The age, BMI, nodule diameter, TG, TC, and blood pressure of the PDCA group and the routine group were statistically analyzed to show that there was no significant difference between them, and the two groups were comparable (*P* > 0.05) (Table 1).

### 3.2. Comparison of Microinflammation Indexes between the PDCA Group and Routine Group

There was no significant difference in CRP, IL-1, TNF-*α*, and IL-6 levels between the two groups before intervention (*P* > 0.05). After that, these levels in the PDCA group were lower than those in the routine group, with statistically significant difference (*P* < 0.05) (Table 2).

### 3.3. Comparison of Nursing Quality of Fistula between the PDCA Group and Routine Group

Before intervention, there was no statistically significant difference in the qualification rate of blood flow, the awareness rate of health education, and the incidence of nursing defects between the two groups (*P* > 0.05). After that, the qualification rate of blood flow and the awareness rate of health education among nurses in the PDCA group were higher than those in the routine group, while the incidence of nursing defect accidents in the PDCA group was lower than that in the routine group, and the differences were statistically significant (*P* < 0.05).  Table 3.

### 3.4. Comparison of Complication Rate between the PDCA Group and Routine Group

Before intervention, there was no significant difference in the complication rate between the two groups (*P* > 0.05). After that, the complication rate of the PDCA group was lower than that of the routine group, and the differences were statistically significant (*P* < 0.05).  Table 4.

### 3.5. Comparison of Theoretical Assessment and Practical Skills Assessment Scores between the PDCA Group and Routine Group of Nursing Staff

After intervention, the theoretical assessment and practical skills assessment scores of the PDCA group were higher than those of the routine group, and the differences were statistically significant (*P* < 0.05) (Table 5).

### 3.6. Comparison of Nursing Satisfaction between the PDCA Group and Routine Group

After intervention, the nursing satisfaction of the PDCA group was higher than that of the routine group, and the differences were statistically significant (*P* < 0.05) (Table 6).

## 4. Discussion

In recent years, the incidence of chronic kidney disease has been increasing. Some patients with chronic kidney disease will gradually aggravate and turn to end-stage renal disease, which requires renal replacement therapy. With the continuous improvement of hemodialysis technology and nursing level, the survival time and quality of life of patients were significantly improved. According to clinical studies, the duration of fistula maintenance in hemodialysis is closely related to surgical skills, vascular conditions, and nursing quality [12, 13].

In recent years, PDCA cycle training mode has been introduced in clinical practice. This method includes random assessment results and regular assessment results, which has the advantages of timely feedback of nursing problems. In addition, it can timely feed back the problems in the nursing process and discuss and correct them, with pertinence and purpose, so that the nursing process is in a virtuous cycle, and the patency rate of patients with arteriovenous fistula can also be improved [14]. In this study, patients were divided into the PDCA group and the routine group, respectively, with PDCA nursing management mode and routine nursing management mode to explore the application of PDCA method in the management of nurses in hemodialysis center and the maintenance effect on internal fistula.

The excessive expression of inflammatory factors such as TNF-*α*, IL-1, and IL-6 in the peripheral blood of MHD patients can stimulate the inflammation of the body and then cause a series of pathological changes. However, in hemodialysis treatment, a puncture surgery (even the repeated puncture in special cases) needs to be done for arteriovenous fistula, causing more chance of contact of the vascular with the outside world, thus leading to the greater probability of infection caused by retrograde blood entry of bacteria and the higher risk of microinflammation reactions [15, 16]. The results of this study showed that there was no significant difference in the complication rate between the two groups before intervention (*P* > 0.05); after intervention, the complication rate of the PDCA group was lower than that of the routine group; there was no significant difference in CRP, IL-1, TNF-*α*, and IL-6 levels between them before intervention (*P* > 0.05). After intervention, the above inflammatory factors in the PDCA group were significantly lower than those in the conventional group. In the implementation of PDCA cycle management mode, nurses pay attention to the observation of patients' blood flow and the blood color in hemodialysis pipeline and can monitor the pulse around the fistula to detect fistula occlusion signs early and give treatment timely. And the measurement of the blood viscosity is beneficial for the timely adjustment of anticoagulant dosage in order to prevent bleeding. The head nurse will formulate nursing goals and implement them in order to reduce the incidence of complications. The head nurse plays a vital role in the whole PDCA model. She should not only hold the monthly discussions which report the problems existing in nursing in the group but also summarize and reflect on the feedback problems and adjust the nursing plan in time [17]. Under the PDCA mode, nurses in the department should formulate targeted nursing measures according to the occurrence of microinflammation and complications and intervene them through planning, doing, checking, and adjusting to effectively reduce the incidence of complications.

The results of this study showed that there was no significant difference in the qualified rate of blood flow, the awareness rate of health education, and the incidence of nursing defect accidents between the two groups before intervention; after that, the qualified rate of blood flow and the awareness rate of health education in the PDCA group were higher than those in the routine group, and the incidence of nursing defects in the PDCA group was lower than that in the routine group. Some studies have shown that PDCA cycle is conducive to building a good relationship between nurses and patients for the better communication; thus, the nursing staff can understand the needs of patients for a better work [18]. Combined with the results of this study, PDCA circulation method enables patients and their families to understand the content of health education for improving their cognition of hemodialysis, which helps patients maintain a good attitude for a better treatment compliance. All of these can prolong the use time of internal fistula and reduce the incidence of nursing defect accidents.

The results of this study showed that after intervention, the scores of theoretical assessment, practical skills assessment, and nursing satisfaction in the PDCA group were significantly higher than those in the routine group. The PDCA method provides patients with more professional and personalized nursing services. Previous studies have shown that dialysis can restore the physiological function of patients to a certain extent, but the changes of the disease itself, complications after treatment, and the costs of treatment affect the quality of patients' life. In this study, the PDCA cycle method was adopted to reduce complications and improve treatment outcomes, which improved the quality of patients' life. In this study, through the PDCA cycle management model, the head nurses in the department coordinated the whole process, formulated the nursing scheme and assessment scheme for clinical practice and theoretical knowledge, developed the corresponding system, completed the training work, and implemented 24-hour continuous nursing. For the improper operation in the whole treatment process, the head nurse gave timely correction. In addition, the head nurse has not regularly inspected the implementation of PDCA cycle management mode to promote the improvement of nursing quality.

In view of the problem that PDCA improves the maintenance effect of internal fistula, it is considered that the nurse has made continuous inspections throughout the treatment period and made emergency treatment plans. In this study, it is found that the inflammatory state will affect the effect of internal fistula. The nursing staff will adjust the nursing plan according to the inflammatory state of the patients and make timely intervention when the internal fistula occlusion and blood viscosity are found. In addition, nurses also require patients and their families to master the knowledge of fistula maintenance and improve their self-observation and nursing ability. When patients are discharged, they can also get self-care at home. The head nurses' meetings are held regularly to explore the problems reflected in the work of the department and adjust the nursing scheme according to the problems of patients and the requirements of patients, so that the medical and nursing scheme is more accurate and humanized. The above measures are conducive to improving the maintenance effect of internal fistula.

The PDCA cycle method clearly reflects the nursing process of evaluation, intervention, and effectiveness evaluation and helps hemodialysis nurses to formulate predictive nursing plans for prediction. The PDCA cycle method integrates assessment, intervention, and evaluation. It can not only discover the common problems of patients and give small group intervention but also take targeted case intervention measures to improve theoretical level and practical skills. This study found that the PDCA method is feasible for maintenance hemodialysis patients.

In the past, the evaluation of the effect of hemodialysis is mostly carried out from the aspects of inflammation and complications [19, 20]. This study uses the PDCA cycle method to effectively improve the professional skills of nurses, improve the qualified rate of blood flow after treatment, improve the awareness rate of health education, reduce the incidence of nursing defects, and improve the quality of care of hemodialysis patients. The sample size selected in this study is small, so further research should consider expanding the sample size and verify the effectiveness of this study through large-capacity sample data.

In summary, the application of the PDCA method in the management of nurses in hemodialysis centers can effectively improve the quality of internal fistula management and the practice and theoretical level of nurses, as well as reduce the microinflammatory state of patients.

## Figures and Tables

**Table 1:** Comparison of baseline data between the PDCA group and routine group.

Group	*n*	Age (years)	BMI (kg/m^2^)	Years of education (years)	Gender (%)		Dialysis time (years)	Primary disease (%)		Fistula location (%)	
					Male	Female		Glomerulus nephritis	Nephrotic syndrome	Left arm	Right arm
PDCA group	45	64.77 ± 7.50	22.63 ± 2.11	7.50 ± 1.64	25 (55.56)	20 (44.44)	2.77 ± 0.68	37 (82.22)	8 (17.78)	21 (46.67)	24 (53.33)
Regular group	45	62.60 ± 7.38	22.48 ± 1.96	7.87 ± 2.01	19 (42.22)	26 (57.78)	2.84 ± 0.70	33 (73.33)	12 (26.67)	26 (57.78)	19 (42.22)
*t*/*χ*^2^		1.383	0.349	-0.957	1.601		-0.481	1.029		1.113	
*P*		0.170	0.728	0.341	0.206		0.632	0.310		0.291	

**Table 2:** Comparison of microinflammation indexes between the PDCA group and routine group($\bar{x}\pm s$).

Group	*n*	CRP(mg/L)		IL-1(ng/mL)		TNF-*α*(pg/mL)		IL-6(pg/mL)	
		Before intervention	Postintervention	Before intervention	Postintervention	Before intervention	Postintervention	Before intervention	Postintervention
PDCA group	45	6.17 ± 1.77	4.03 ± 1.36	84.39 ± 9.76	75.40 ± 7.70	73.78 ± 10.60	66.19 ± 8.42	42.84 ± 7.37	35.80 ± 6.61
Regular group	45	6.33 ± 1.80	5.14 ± 1.52	86.20 ± 10.54	81.00 ± 8.95	72.14 ± 9.62	70.37 ± 8.58	41.90 ± 7.55	38.92 ± 6.38
*t*		-0.425	-3.651	-0.845	-3.182	0.769	-2.333	0.598	-2.278
*P*		0.672	0.000	0.400	0.002	0.444	0.022	0.552	0.025

**Table 3:** Comparison of nursing quality of internal fistula between the PDCA group and routine group ($\bar{x}\pm s$).

Group	*n*	Blood flow pass rate		Awareness rate of health education		Nursing deficiency incident	
		Before intervention	After intervention	Before intervention	After intervention	Before intervention	After intervention
PDCA group	45	38 (84.44)	44 (97.78)	27 (60.00)	42 (93.33)	6 (13.33)	1 (2.22)
Regular group	45	35 (77.78)	36 (80.00)	31 (68.89)	37 (82.22)	8 (17.78)	6 (13.33)
*χ* ^2^		0.653	7.200	0.776	2.589	0.338	3.873
*P*		0.419	0.001	0.378	0.108	0.561	0.049

**Table 4:** Comparison of complication rate between the PDCA group and routine group.

Group	*n*	Incidence of subcutaneous hematoma	Incidence of fistula blockage	Infection rate	Steal syndrome	Swollen hand syndrome	Complication rate (%)
PDCA group	45	0	1	1	0	1	3 (6.67)
Regular group	45	3	2	2	1	2	10 (22.22)
*χ* ^2^							4.406
*P*							0.036

**Table 5:** Comparison of theoretical assessment and practical skills assessment scores of nursing staff ($\bar{x}\pm s$, scores).

Group	*n*	Theoretical assessment	Practical skills
PDCA group	45	91.63 ± 3.87	90.08 ± 4.73
Regular group	45	87.85 ± 5.03	87.64 ± 4.80
*t*		3.995	2.429
*P*		0.000	0.017

**Table 6:** Comparison of meeting satisfaction between the PDCA group and conventional group (*n* (%)).

Group	*n*	Very satisfied	Satisfy	Generally	Dissatisfied
PDCA group	45	28 (62.22)	15 (33.33)	2 (4.44)	0 (0.00)
Regular group	45	16 (35.56)	22 (48.89)	6 (13.33)	1 (2.22)
*Z*		-2.698			
*P*		0.007			

## Data Availability

The raw data supporting the conclusions of this article will be made available by the authors, without undue reservation.
